RETRACTED

# The proto-oncogene *c-src* is involved in primordial follicle activation through the PI3K, PKC and MAPK signaling pathways

**DOI:** 10.1186/1477-7827-10-58

**Published:** 2012-08-20

**Authors:** Xiao-Yu Du, Jian Huang, Liang-Quan Xu, Dan-Feng Tang, Lei Wu, Li-Xia Zhang, Xiao-Ling Pan, Wei-Yun Chen, Li-Ping Zheng, Yue-Hui Zheng

**Affiliations:** 1 Medical Experimental Teaching Department, Nanchang University, Nanchang, 330006, China; 2 Department of Physiology Reproduction, Medical College of Nanchang University, Nanchang, 330006, China; 3 Department of Academic Journal, Nanchang University, Nanchang, 330006, China

## Abstract

**Background:**

*C-src* is an evolutionarily conserved proto-oncogene that regulates cell proliferation, differentiation and apoptosis. In our previous studies, we have reported that another proto-oncogene, *c-erbB*_*2*_, plays an important role in primordial follicle activation and development. We also found that *c-src* was expressed in mammalian ovaries, but its functions in primordial follicle activation remain unclear. The objective of this study is to investigate the role and mechanism of *c-src* during the growth of primordial follicles.

**Methods:**

Ovaries from 2-day-old rats were cultured *in vitro* for 8 days. Three *c-src*-targeting and one negative control siRNA were designed and used in the present study. PCR, Western blotting and primordial follicle development were assessed for the silencing efficiency of the lentivirus *c-src* siRNA and its effect on primordial follicle onset. The expression of *c-src* mRNA and protein in primordial follicle growth were examined using the PCR method and immunohistochemical staining. Furthermore, the MAPK inhibitor PD98059, the PKC inhibitor Calphostin and the PI3K inhibitor LY294002 were used to explore the possible signaling pathways of *c-src* in primordial folliculogenesis.

**Results:**

The results showed that Src protein was distributed in the ooplasmic membrane and the granulosa cell membrane in the primordial follicles, and *c-src* expression level increased with the growth of primordial follicle. The *c-src* -targeting lentivirus siRNAs had a silencing effect on *c-src* mRNA and protein expression. Eight days after transfection of rat ovaries with *c-src* siRNA, the GFP fluorescence in frozen ovarian sections was clearly discernible under a fluorescence microscope, and its relative expression level was 5-fold higher than that in the control group. Furthermore, the *c-src*-targeting lentivirus siRNAs lowered its relative expression level 1.96 times. We also found that the development of cultured primordial follicles was completely arrested after *c-src* siRNA knockdown of *c-src* expression. Furthermore, our studies demonstrated that folliculogenesis onset was inhibited by Calphostin, PD98059 or LY294002 treatment,but none of them down-regulated *c-src* expression. In contrast, the expression levels of p-PKC, p-ERK1/2 and p-PI3K in the follicles were clearly decreased by *c-src* siRNA transfection. Correspondingly, both Calphostin and LY294002 treatment resulted in a decrease in the p-PKC level in follicles, but no change was observed in the PD98059 group. Finally, LY294002 treatment decreased the p-PI3K expression level in the follicles, but no changes were observed in the PD98059 and Calphostin groups.

RETRACTED

**Conclusions:**

*C-src* plays an important role in regulating primordial follicle activation and growth via the PI3K-PKC- ERK1/2 pathway.

## Introduction

Oocytes are surrounded by somatic cells in the ovaries of newborn mammals. In rats, during the first 3 days after birth, the primordial follicles are assembled and remain developmentally arrested thereafter until the primary follicles are formed later [1]. The primordial follicle growth signals the transition of the primordial follicle from quiescence to the next growth state—the primary follicle stage. As the process commences, the oocytes begin to grow and the granulosa cells around the oocyte become cubiform and proliferate rapidly. When the cubiform granulosa cells surrounding the growing oocytes reach more than one layer, the follicle become the secondary follicle [2]. This progress requires a coordinated interaction of events, such as cell cycle progression, apoptosis, and differentiation of pluripotent somatic cells into the granulosa cell lineage. Although the exact factors and mechanisms that regulate folliculogenesis initiation remain elusive, the accumulated evidence suggests that the early growth stage of follicle development is not dependent on the gonadotropins but is mainly controlled by a combination of local paracrine factors within the ovaries. Some factors, such as stem cell factor (SCF), epidermal growth factor (EGF), basic fibroblast growth factor (bFGF), leukemia inhibitory factor (LIF), nerve growth factor (NGF), bone morphogenic protein (BMP), growth differentiation factor 9 (GDF-9) and insulin-like growth factor (IGF), promote the development of the primordial follicles. Other factors, such as AMH, E_2_ and P, inhibit primordial follicle development [3-6]. Although we still poorly understand at the molecular level how these factors regulate primordial follicle development, successful activation of follicle growth must involve genetic networks both in germ and somatic cells. In recent years, genetic factors have received increasing attention as determinants of primordial follicle onset [7-11]. In a recent study, we have showed that the mRNA of another Proto-oncogene, *c-erbB*_*2*_, is expressed in the primordial follicle, and ablation of *c-erbB*_*2*_ in neonatal rat ovaries results in excessive inhibition of primordial follicles [12], which demonstrates that *c-erbB*_*2*_ plays an important role in regulating primordial follicle onset. In addition to the evidence from our previous studies that *c-src* mRNA is expressed in mammalian ovaries, primordial follicle growth was retarded and the number of mature follicles was significantly reduced in *c-src* knock-out mice [13,14]. Based on this finding, it is tempting to speculate that *c-src* might play an important role in regulating primordial follicle onset as well.

RETRACTED

The proto-oncogene *c-src,* an evolutionarily conserved proto-oncogene and the first carcinoma gene to be discovered in cells by Bioshop *et al.* in 1976, is widely expressed in yeast, Drosophila and vertebrates, including humans. *c-src* participates in the regulation of cell growth, development, differentiation and other biological functions. Src protein was the first member of the Src protein family kinases (SFKs) to be identified, and it is a non-receptor tyrosine protein kinase. During the oocyte maturation process, phosphorylated SFKs and non-phosphorylated SFKs are concentrated in the nucleus and the cortical region of the oocytes before germinal vesicle breakdown (GVBD). Once GVBD occurs, the activated SFK is distributed throughout the oocytes [15-17]. These findings suggest that *c-src* plays an important role in oocyte maturation. However, whether *c-src* and Src protein are expressed during primordial follicle growth and what roles they play in this process have not been reported.

A variety of signaling pathways, including the MAPK and PKC pathways, are involved in the activation of the growth of primordial follicles [18-21]. Signaling pathways, such as the PI3K and mTORC1 pathways, regulate the activation of primordial follicles and the early development of ovarian follicles [7,11]. It is possible that Src protein and the three intracellular signaling proteins (MAPK, PKC, PI3K) are inextricably linked. Both PKC isozymes and Fyn protein kinase exist in mammalian follicles, and PKC might induce the activation of eggs [22,23]. PP2, an inhibitor of Src protein, hindered the phosphorylation of PI3K and Akt [24-26]. In this study, we will explore the possible signaling roles of *c-src* in primordial follicle initiation in the context of other canonical signaling pathways.

## Methods

### Animals and reagents

The animal use was approved by the Committee of Nanchang University for Animal Research. Two-day-old Sprague Dawley rats (weight approximately 4-6g) were used for all the experiments. The immunohistochemical kit was purchased from ZhongShan Co., Ltd. (Beijing, China). The monoclonal antibodies against Src protein, PD98059 (a MAPK inhibitor), Calphostin (a PKC inhibitor) and LY294002 (a PI3K inhibitor), β-actin and Lipofectamine2000 were purchased from Sigma (St. Louis MO). The EASY siRNA kit was purchased from Genechem Co., Ltd. (Shanghai, China) and the lentivirus-packaged siRNA was prepared by Genechem Co., Ltd. (Shanghai, China).

RETRACTED

### Designation, construction and transfection of lentivirus c-src siRNA

In brief, three *c-src*-targeting oligonucleotides (siRNA1, siRNA2, siRNA3, targeting to the *c-src* gene NM_031977) were designed, and another was used as the negative control (no siRNA). Transfection was performed according to the instructions provided with Lipofectamine2000. The ovaries were cultured in 24-well plates. After 36 h, they were transferred to serum-free culture solutions with 40 pmol/l of siRNA1, siRNA2 or siRNA3. After 12 h of transfection, the medium was replaced with fresh medium containing no siRNA, and the ovaries were cultured for an additional 8 days. Furthermore, the specimen with the interference effects were evaluated by RT-PCR and western blotting, and the siRNA that produced the most effective knockdown was synthesized and packed into a lentiviral vector (1.5 × 10^9^IU/ml). The best interference effect for *c-src* siRNA was as follows: sense, 5’-CACUACAAGAUCCGGAAACtt-3’, antisense, 5’-GUUUC CGGAUCUUG UAGUGtt-3’.

### Culture of neonatal rat ovaries and experimental protocol

Ovaries from postnatal Day 2 Sprague–Dawley rat pups were cultured as previously described [18]. For the *in vitro* studies, the ovaries were divided into three groups: *c-src* siRNA group (lentiviral *c-src* siRNA; *c-src* siRNA), negative control group (blank vector; lentivirus without siRNA), and blank control group (*c-src*-non-targeting oligonucleotides). The medium was replaced every 48 h with fresh medium containing no siRNA, and the ovaries were cultured for 8 days. To determine the upstream and downstream relationships between *c-src*, MAPK, PKC and PI3K, the ovaries were challenged with PD98059 (5 × 10^-2^ mmol/L), Calphostin (5 × 10^-4^ mmol/L) or LY294002 (5 × 10^-2^ mmol/L). After termination, the ovaries were processed for morphometric evaluation of follicular development by the detecting levels of mRNA, immunohistochemistry and western blotting analysis.

### Histological morphometric evaluation of folliculogenesis

Ovaries from 2-day-old rats were collected fresh or cultured for 4 and 8 days (ovaries were cultured with/without inhibitors and lentiviral *c-src* siRNA), with 16 ovaries in each group. Fresh ovaries were fixed in Bouins solution for 1–2 h, embedded in paraffin, sectioned (3-5 × 10^-3^ mm) and stained with hematoxylin and eosin. The number of follicles at each developmental stage was counted in two serial sections from the largest cross-section through the center of the ovary. Typically, two ovaries were included in each treatment group as replicates, and 150–200 follicles were present in each ovary cross-section. The experiments were repeated three times (therefore, n = 6 for each treatment group). Primordial follicles are known to consist of one oocyte that is partially or completely encapsulated by flat squamous pregranulosa cells. Developing follicles contain successively more cuboidal granulosa cells in the layers around the oocyte.

RETRACTED

### Immunohistochemistry to determine the localization of src protein

Paraffin-embedded rat ovaries were sectioned to 3-5 × 10^-3^ mm and set in the oven at 60°C for half an hour. The tissue sections were deparaffinized, and the endogenous peroxidase activity was quenched with 3% H_2_O_2_ in methanol. Following rehydration, nonspecific binding was blocked with binding liquid, and the sections were then incubated for 2 h with monoclonal antibodies against the Src protein at 37°C. Following extensive washing with PBS, the tissue sections were incubated with a biotin-conjugated secondary antibody at 37°C for 20 min. After washing with PBS, the tissue sections were quenched with HRP-working liquid for 20 min at 37°C to detect and bind to the secondary antibodies. After treatment with DAB, the tissue sections were counterstained with hematoxylin. Following dehydration, hyaline, drying and finalizing, the sections were set under an inverted microscope for imaging. We used PBS instead of monoclonal antibodies toward Src protein as a negative control.

### Quantitative reverse transcriptase-polymerase chain reaction (RT-PCR) to determine the levels of c-src and β-actin mRNA

Expression of mRNA for *c-src* was assayed by RT-PCR. Ovaries from the same culture wells described above were pooled to prepare a single RNA sample. The ovaries that had been cultured with inhibitors and a reorganizing lentivirus were also assayed by RT-PCR. RNA was extracted using the Trizol reagent (Sigma, St. Louis, MO). Total RNA from each sample was reverse transcribed into cDNA using a standard oligo-dT RT protocol. cDNA samples were used as a template for polymerase chain reaction (PCR) analysis. The 2 × EasyTaq PCR Supermix kit (TRansGen Biotec) was used according to the manufacturer’s instructions. The *c-src* primers were as follows: forward sequence: 5’-CAT CCA AGC CTC AGA CCC A-3’, reverse: 5’-TGA CAC CAC GGC ATA CAG C-3’. The housekeeping reference gene β-actin primers were as follows: forward: 5’-ACA CTG TGC CCA TCT ACG AGG-3’, reverse: 5’-AGG GGC CGG ACG CGT CAT ACT- 3’. The samples were heated to 94°C for 4 min and then submitted to 35 cycles of 95°C for 45 sec, 55°C for 45 sec and 72°C for 1 min, and followed by an extension step at 72°C for 7 min. The fluorescent detection data for *c-src* mRNA were analyzed and normalized relative to the β-actin mRNA levels. The identities of the RT-PCR products were confirmed by direct sequencing (Shanghai Sangon Biological Engineering Technology & Services Co. Ltd.). All experiments were repeated at least three times.

RETRACTED

### Real-time PCR determination of the levels of c-src and β-actin mRNA

To analyze *c-src* mRNA levels, total RNA was extracted from cultured rat ovaries and used as a template for cDNA synthesis using oligo (dT) primers and the SuperscriptIII kit (Invitrogen, CA). Total DNA was extracted from the rat ovaries to assess GFP DNA levels. Real-time quantitative PCR was performed using the ABI Prism 7500 detection system (PE Applied Biosystems, Foster City, CA) with the SYBR green DNA detection kit (Applera, NY). The expression levels of the house keeping gene encoding β-actin were also quantified using 50 ng of cDNA. The relative mRNA values were determined and used for normalization. All experiments were repeated at least three times. The PCR primers for *c-src* were as follows: forward primer: 5'- GGACAGTGGCGGATTCTACATC-3', reverse primer: 5'- AGCTGCTGCAGGCTGTTGA-3'. The reaction conditions were as follows: 95°C for 30 sec, 95°C for 5 sec, 60°C for 60 sec for a total of 45 cycles. The amplicon size was 57 bp. The PCR primers for β-actin were as follows: forward primer: 5'- TTCAACACCCCAGCCATGT-3', reverse primer: 5'- CAGAGGCATACAGGGACAACAC-3', and the amplicon size was 58 bp. The PCR primers for GFP were as follows: forward primer: 5'-TGCTTCAGCCGCTACCC-3', reverse primer: 5'-CTTGCCGTAGTTCCACTTGA-3'. The reaction conditions for GFP PCR were as follows: 95°C for 15 sec, 95°C for 5 sec, 60°C for 30 sec for a total of 45 cycles.

### Detection and quantification of src protein, p-ERK^1^/_2_, p-PKC and p-PI3K by Western blotting analysis

Ovaries that had been cultured for 8 days were pooled to produce a single protein sample. The levels of Src, p-ERK1/2, p-PKC, p-PI3K or β-actin protein in ovaries that had been cultured with inhibitors and a reorganizing lentivirus were assayed by western blotting.

Tissue protein extracts were electrophoretically separated under reduced conditions using NuPAGE 7.5–10% Bis-Tris gels (Invitrogen; Paisley, UK). Standard Mark (Invitrogen) was used as the molecular weight standard. The proteins were then electrotransferred to nitrocellulose membranes (BIORAD; Munich, Germany, 4°C, 230 mA, 1.5 h), and the immunoblots were subsequently blocked for 2 h at room temperature in TBST (TBS containing 0.1% Tween 20) containing 2.5% BSA. The membranes were incubated overnight at 4°C with antibodies against Src, p-ERK1/2, p-PKC, p-PI3K or β-actin (1:200). The β-actin bands were used as an internal control for equal loading. After rinsing with TBST, the membranes were incubated for 2 h at 37°C with horseradish peroxidase-conjugated anti-rabbit or anti-mouse secondary antibodies (1:500). Finally, the membranes were treated with ECL in a darkroom, exposed, developed and fixed and imaged. We analyzed the images with the Gel image analysis system.

RETRACTED

### Fluorescence imaging

After 8 days of culture with the lentivirus, the rat ovaries were removed and cut into 5-μm-thick serial sections. GFP fluorescence was observed using a fluorescence microscope (Leica, Germany).

### Statistics

To evaluate follicle development, three ovaries from different rats were cultured for each treatment group, and the cultures were repeated at least twice. For immunohistochemistry, we used one ovary per group, and the cultures were repeated three times. For RNA and protein preparation, three ovaries per group were cultured and then pooled into one sample. The cultures were repeated three times. All data were presented as the means ± SEM and analyzed by ANOVA and Duncan’s new multiple range tests. *p <* 0.05 was considered significantly different.

## Results

### Src protein expressed in rat ovaries during primordial follicle culture

The expression of *c-src* protein in the ovaries during primordial follicle growth was examined by immunohistochemistry analysis. Src protein was detected in the oocytes and granulosa cells of primordial follicles and primary follicles. During the development of the follicles, the expression of Src protein increased correspondingly (*p* < 0.01) (Figure 1).

**Figure 1:** **Expression of Src protein in rat ovaries during the activation and growth of primordial follicle were examined by immunohistochemistry analysis.** Src protein expression in the oocyte and granulosa cell membrane of primordial and primary follicles (red arrows) is shown in **A**, **B** and **C** (which represent ovaries cultured *in vitro* for 0, 4 and 8 days, respectively). During the development of the follicles, the expression of Src protein increased corresponding. The negative controls are shown in **D**, **E** and **F** (which represent ovaries cultured *in vitro* for 0, 4 and 8 days, respectively).

RETRACTED

### siRNA knockdown of c-src mRNA and protein suppresses primordial follicle development

The specificity of the *c-src* siRNA effect was verified by examining the levels of *c-src* mRNA and protein in ovaries exposed to *c-src* siRNA. Compared with blank control and negative control, siRNA specifically and appreciably reduced the levels of *c-src* mRNA (Figure 2) and *c-src* protein (Figure 3) in the ovaries. When the ovaries were cultured with lentivirus packaging siRNA particles, the β-actin mRNA and protein were not affected by any treatment, suggesting the specificity of the *c-src* siRNA (Figure 2, Figure 3).

**Figure 2:** **The silencing efficiency of the lentivirus after transfection.A**, *c-src* mRNA in ovaries 8 days after lentivirus transfection and a semiquantitative assay of the *c-src* mRNA levels 8 days after lentiviral transfection from six different replicates. **B**, Real-time PCR was used to analyze the relative *c-src* mRNA (*c-src* mRNA/β-actin mRNA). Blank control corresponds to the group that was transfected with c-src-non-targeting oligonucleotides, negative control corresponds to the group that was transfected with a blank vector (lentivirus without siRNA), and c-src siRNA corresponds to the group with the lentivirus packaging *c-src* siRNA. The data are presented as the means ± SEM (n = 3). **P<0.01 compared with the negative control group.

**Figure 3:** **The silencing efficiency of the lentivirus after transfection.A**, *c-src* protein in the ovaries 8 days after lentivirus transfection. **B**, Semiquantitative results of western blotting from three different replicates. Blank control corresponds to the group with *c-src*-non-targeting oligonucleotides, negative control corresponds to the group with blank vector (lentivirus without siRNA), and *c-src* siRNA corresponds to the group with lentivirus packaging *c-src* siRNA. The data are presented as the means ± SEM (n = 3). **P<0.01 compared with the negative control group.

The delivery efficiency was measured by fluorescence imaging. Eight days after transfection of the rat ovaries with *c-src* siRNA, the GFP fluorescence of frozen ovarian sections was clearly observed under a fluorescence microscope. Furthermore, the GFP DNA level increased significantly, and its relative expression level was 5.07 times higher than that in the control group, and the *c-src* siRNAs lowered the GFP DNA relative expression level 1.96 times. These results demonstrated that the lentivirus was successfully delivered to the ovarian tissue by *in vitro* organ culture (Figure 4).

**Figure 4:** **The delivery efficiency of the lentivirus after transfection.A**,The GFP fluorescence of frozen ovarian sections 8 days after lentivirus transfection. **B**, Semiquantitative assay of the relative level of GFP DNA 8 days after lentivirus transfection from six different replicates. Blank control corresponds to the group with *c-src*-non-targeting oligonucleotides, negative control corresponds to the group with blank vector (lentivirus without siRNA), and *c-src* siRNA corresponds to the group with lentivirus packaging *c-src* siRNA. The data are presented as the means ± SEM (n = 3). ** *P<*0.01 compared with blank control; Δ *P<*0.05 vs. negative control.

RETRACTED

To clarify whether *c-src* was involved in activation of the growth of primordial follicles, we transferred *in vitro* synthesized siRNAs into the newborn rats' ovaries to examine the effect of *c-src* on primordial follicle development. Neonatal rat ovaries cultured for 8 days in the blank control group contained approximately 35% primordial follicles, and the percentage was not altered when the ovaries were exposed to the negative control. *c-src* siRNA significantly retarded the development of primordial follicles, as approximately 64% of the primordial follicles remained in the siRNA-treated ovaries. Together with the evidence of constitutive Src distribution in the primordial follicles, the results of the effect of *c-src* inhibition by siRNAs on primordial follicle growth suggested that *c-src* might be essential for primordial follicle development (Figure 5).

**Figure 5:** **Effect of*c-src*siRNA on the activation of primordial follicle growth.A**, Ovaries were cultured for 8 days with the indicated treatments: blank control, negative control, 100 μmol/L siRNA targeting *c-src*. Ovarian sections were stained with hematoxylin and eosin to show the follicles at different developmental stages. Scale bar: 20 μm. HE staining X400 **B**, The number of follicles was counted in serial cross-sections. The percentage of the number of each category over the total number was plotted. The data are presented as the means ± SEM. Bars with different superscripts are statistically different (*P<*0.01). Blank control corresponds to the group with *c-src*-non-targeting oligonucleotides, the negative control corresponds to the group with blank vector (lentivirus without siRNA), and *c-src* siRNA corresponds to the group with lentivirus packaging *c-src* siRNA. The data are presented as the means ± SEM (n = 3). **P<0.01 compared with negative control group.

### The effect of c-src on primordial follicle development involving the MAPK, PKC and PI3K signaling pathway

PD98059, Calphostin and LY294002 are widely used as MAPK, PKC and PI3K inhibitors, respectively. After culturing neonatal rat ovaries for 8 days, each of these compounds inhibited primordial follicle development significantly (Figure 6). These results suggest that the MAPK, PKC and PI3K signaling pathways are vital to primordial follicle development. We added PD98059, Calphostin and LY294002 to the culture solution and collected specimens to detect *c-src* mRNA levels by real time-PCR and Src protein abundance by western blotting. The development of primordial follicles was observed by hematoxylin/eosin (HE) staining. We found that, compared with the blank group, the *c-src* mRNA and Src protein levels in each inhibitor group were not reduced (P > 0.05) (Figure 7, Figure 8). Treatment of cultured primordial follicles with the *c-src* siRNA not only suppressed the levels of src protein, but also the phosphorylation of ERK1/2, PKC and PI3K (Figure 8), suggesting that the activation of MAPK, PKC and PI3K in primordial follicle is downstream of the *c-src* proto-oncogene. In addition, as shown in Figure 8, we found that p-ERK1/2 in the follicles decreased after PD98059, Calphostin and LY294002 treatment, suggesting that activation of MAPK in the follicles is downstream of PKC and PI3K. The levels of p-PKC in the follicles decreased after Calphostin and LY294002 treatment, but no change was observed after treatment with PD98059, suggesting that activation of PKC in the follicles is downstream of PI3K and upstream of MAPK. The levels of p-PI3K in the follicles decreased after LY294002 treatment, but no changes were detected in the PD98059 and Calphostin groups, suggesting that activation of PI3K in the follicles is upstream of MAPK and PKC. Therefore, we conclude that the effect *c-src* on primordial follicle development is involved in the MAPK, PKC and PI3K signaling pathways, and the direction of the cascade may be *c-src* → p-PI3K → p-PKC → p-ERK1/2 (Table 1 and Figure 9).

RETRACTED

**Figure 6:** **Effect of PD98059, Calphostin and LY294002 on the activation of primordial follicle growth.A**, Ovaries were cultured for 8 days with treatments: blank control, PD98059(5 × 10^-2^ mmol/L), Calphostin (5 × 10^-4^ mmol/L)and LY294002(5 × 10^-2^ mmol/L). Ovarian sections were stained with hematoxylin and eosin to show the follicles at different developmental stages. Scale bar: 20 μm. HE staining X400 **B**, The number of follicles was counted in serial cross-sections. ** *P<*0.01 vs. blank control.

**Figure 7:** **Effect of the MAPK inhibitor PD98059, the PKC inhibitor Calphostin and the PI3K inhibitor LY294002 on the expression of*c-src*mRNA.A**, The expression of *c-src* mRNA (250 bp) in the ovaries by RT-PCR and semiquantitative analysis of the RT-PCR results. **B**, Real-time PCR was used to analyze the relative levels of *c-src* mRNA (*c-src* mRNA/β-actin mRNA). The data are presented as the means ± SEM (n = 3).

**Figure 8:** **The expression of Src, p-ERK1/2, p-PKC and p-PI3K protein after*c-src*siRNA, PD98059, Calphostin and LY294002 treatment, respectively.A**,The expression of Src, p-ERK1/2, p-PKC and p-PI3K protein in the ovaries detected by western blotting. **B**, The expression of Src protein according to a semiquantitative analysis of the western blot result. **C**, The expression p-ERK1/2 protein according to a semiquantitative analysis of the western blot result. **D**, The expression of p-PKC protein according to a semiquantitative analysis of the western blot result. **E**, The expressions of p-PI3K protein by semiquantitative analysis of the western blot result. Blank control corresponds to the group transfected with negative control siRNA. The data are presented as the means ± SEM (n = 3). ** *P<*0.01 vs. blank control group.

**Table 1:** ***C-src*involved in p-PI3K, p-PKC and p-ERK1/2 signal cascades in primordial follicle development**

**Treatment**	**The relationship and the changes**				
	***c-src*→**	**p-PI3K→**	**p-PKC→**	**p-EPK1/2→**	**follicle growth**
*c-src* siRNA	↓	↓	↓	↓	↓
LY294002	-	↓	↓	↓	↓
Calphostin	-	-	↓	↓	↓
PD98059	-	-	-	↓	↓

↓ stands for down regulation of expression; -symbols for no change.

**Figure 9:** ***C-src*regulating primordial follicle activation and growth through PI3K → PKC → MAPK signaling pathway**

## Discussion

### Location and analysis of src mRNA and protein in primordial follicles

Our PCR results showed that *c-src* mRNA was present in SD rat primordial follicles, which was confirmed by sequence comparison with GeneBank. Our immunochemical results confirmed that Src protein mainly localized in the oocyte membrane and granulosa cell membrane in the primordial follicles of neonatal SD rats. Src protein increased during the development of primordial follicles *in vitro*. Previous studies have shown that the egg cortical region is rich in cytoskeletal structures such as actin, microtubules, microfilaments and so on [13]. The different subcellular localization of SFKs might be related to the regulation of intracellular activities, such as mitosis, the rearrangement of the cytoskeleton, and trans-membrane exchange of substances [17]. Src protein, which is also present in the granulosa cell cytoplasm, might be involved in other cytoskeletal activities, especially in terms of granulosa cell-oocyte interaction. However, the finding that the expression of Src protein increased with an increasing culture duration indicated that the activity of *c-src* increased with the development of primordial follicles. In this study, whether the activity of Src protein increased was unclear. Additionally, further examination of whether the crosstalk between the oocytes and the granulosa cells affects the dynamic localization of Src protein in primordial follicles is needed.

RETRACTED

### The effect of c-src on primordial follicles and its mechanism of action

Cultured ovarian tissue that was transfected with siRNA1 packaged into a lentiviral vector had decreased levels of *c-src* mRNA and Src protein compared with the control group. The ovarian HE staining demonstrated that the proportion of primordial follicles compared with total follicles increased in the transfected group compared with the control group, demonstrating the inhibitory effect of *c-src* siRNA1 on primordial follicle development. We conjectured that the activity of *c-src* may be essential for promoting the development of primordial follicles.

*c-src* SH2 structural domain binds to Tyr527 at its C’ end (or terminal), and then Tyr57 is phosphorylated by the protein tyrosine kinase C-terminal Src kinase (CSK), which in turn causes the molecular structure to transform, preceding the inhibition of the activity center of the *c-src* kinase [27-29]. The dephosphorylation of Tyr572 can reactivate *c-src*. Once *c-src* kinase is released from its inhibited status, a key Tyr residue inside the PTK functional domain would be phosphorylated due to the activation of PTK. Inter-activation between CSK’s homolog domain SH2/SH3 with certain proteins causes self-phosphorylation of the Tyr residues in the catalytic region of the Src-family protein tyrosine kinases (SFKs), which in turn activates SFK [30]. Talmor-Cohen et al. [13] found that the fusion of rat oocytes and sperm triggers SFK activation, which induces calcium release via the PLC-IP3 pathway and the resumption meiosis. Meng et al. [17] found that transfection of *c-src* siRNA into mouse oocytes before GVBD could reduce the resumption of meiosis by more than 50% compared with controls, similar to the effect of a *c-src* inhibitor.

SFKs are found in rat and mouse oocytes, and they have a role in regulating oocyte maturation [17]. The specific inhibitor of PP2 could decrease the rate of GVBD, which further implies that SFK is independent of mouse oocyte meiosis resumption [31]. SKF maintained its kinase activity by binding to the cell inner membrane through an N-terminal membrane-bound sequence that was covalently linked to myristic acid [32]. However, the execution of the SFK’s functions in oocytes might be related to cytoskeleton microfilaments and microtubules [17]. We conjectured that Src protein might be primarily synthesized in oocytes and granulosa cells and function as a regulator of the activation of primordial follicles via its N-terminal membrane-binding sequence and by mediating the cytoskeletal interactions between granulosa cells and oocytes. We also found that Src protein levels increased over time during culture, indicating that the activity of *c-src* might be elevated during the development of primordial follicles. Thus, we further presumed that endogenous factors inside primordial follicles, such as EGF, may bind to the SH2 structural domain of the Src protein. Alternatively, some factors (e.g., PI3K) produced during the development of the primordial follicle may bind to the SH3 structural domain of Src and caused SH3 to bind to the SH2 structural domain, or SH3 may directly bind to the SH2 structural domain of the Src protein. The exact mechanism of Src protein activation remains to be elucidated.

RETRACTED

### Src protein in primordial follicle development and the PI3K, PKC and MAPK signaling pathways

Many studies have shown that SFK can be activated by growth factors, integrin, superoxide and UV rays. Many growth factors, such as PDGF, FGF, EGF, are upstream activators of the Src protein, not only activating the Src protein but also resulting in ovum activation [30]. The activated SFKs promote the translocation of γ site-phosphates of adenosine triphosphate (ATP) to tyrosine residues in the corresponding target proteins, thus activating the target proteins to a further transmit the signal. Hindering the activity of Src kinase inhibits the activity of MAPK in granulosa cells [33]. The inhibition of mouse oocyte GVBD is due to the activation of PKCα, which may be involved in the regulation of chromatin condensation and nuclear envelope assembly as well as other cellular events during the process of oocyte maturation [15,22]. In mice, rats and other animal oocytes, it has been found that the inhibition of PKC activity in GV stage oocytes and blockade of GVBD also inhibit the activation of MAPK. After its activation, PKC may participate in other functions by inhibiting the upstream molecules of MAPK. However, MAPK is not necessary for GVBD to occur, and PKC may also regulate GVBD through cAMP [16,34]. The secretion of granulosa cells may be mediated by Ca^2+^ release or PKC activation, while SKF can activate PKC by producing DAG, causing a subsequent signaling cascade [13]. *pten* is the inhibitory regulating gene of PI3K. Reddy *et al.* found that the number of primordial follicles in the ovaries was greatly reduced in *pten-*knockout mouse, which led to premature activation of primordial follicles and premature depletion of the follicle reserve, similar to *Foxo3a*–knockout mice. Their findings indicate that *pten* plays an important role in the regulation of premature ovarian failure; meanwhile, the oocyte inhibits follicle activation [8,11].

RETRACTED

Our results showed that the maturity of primordial follicles was not only dependent on the activation of Src protein, but also required the involvement of ERK1/2, PKC and PI3K signaling pathways in primordial follicles. ERK1/2, PKC and PI3K may positively regulate the maturation of primordial follicles. We speculated that Src protein, along with ERK1/2, PKC and PI3K, form a complex signaling network that regulates the development of primordial follicles. The putative signaling cascade is triggered by PI3K, which in turn activates PKC and ultimately causes the activation of MAPK activation.

According to a new study [8], many genes, such as *pten, Tsc1, Tsc2, Foxo3a, p27*, are involved in the silencing and activation of primordial follicles. A better understanding of these signaling pathways and the genetic networks that orchestrate primordial follicle development will be helpful for uncovering the mechanisms underlying many disease conditions, such as female sterility, premature ovarian failure (POF), polycentric ovary disease syndrome (PCOS), and ovarian cancers.

## Conclusions

*C-src* play an important role in regulating primordial follicle activation and growth through the PI3K-PKC-ERK1/2 signaling pathway.

## Competing interests

The authors declare that they have no competing interests.

## Authors’ contributions

DXY, HJ, TDF, XLQ and WL carried out all the experiments. ZYH, DXY, HJ, TDF, XLQ, WL, ZLP, PXL and CWY performed the statistical analysis and drafted the paper. ZYH and ZLP designed the study and amended the paper. All authors read and approved the final manuscript.

## References

[B1] HirshfieldANDevelopment of follicles in the mammalian ovaryInt Rev Cytol199112443101200191810.1016/s0074-7696(08)61524-7

[B2] McNattyKPFidlerAEJuengelJLQuirkeLDSmithPRHeathDALundyTO'ConnellATisdallDJGrowth and paracrine factors regulating follicular formation and cellular functionMol Cell Endocrinol2000163112010.1016/S0303-7207(99)00235-X10963868

[B3] ParrottJASkinnerMKKit-ligand/stem cell factor induces primordial follicle development and initiates folliculogenesisEndocrinology19991404262427110.1210/en.140.9.426210465300

[B4] WangCRoySKExpression of growth differentiation factor 9 in the oocytes is essential for the development of primordial follicles in the hamster ovaryEndocrinology2006147172517341638486610.1210/en.2005-1208

[B5] SkinnerMKRegulation of primordial follicle assembly and developmentHuman Reprod20051146147110.1093/humupd/dmi02016006439

[B6] KezelePRSkinnerMKRegulation of ovarian primordial follicle assembly and development by estrogen and progesterone: endocrine model of follicle assemblyEndocrinology20031443329333710.1210/en.2002-013112865310

RETRACTED

[B7] LiuKRajareddySLiuLJagarlamudiKBomanKSelstamGReddyPControl of mammalian oocyte growth and early follicular development by the oocyte PI3 kinase pathway: new roles for an old timerDev Biol200629911110.1016/j.ydbio.2006.07.03816970938

[B8] ReddyPLiuLAdhikariDJagarlamudiKRajareddySShenYDuCTangWHämäläinenTPengSLLanZJCooneyAJHuhtaniemiILiuKOocyte-specific deletion of Pten causes premature activation of the primordial follicle poolScience200831961161310.1126/science.115225718239123

[B9] ReddyPAdhikariDZhengWLiangSHämäläinenTTohonenVOgawaWNodaTVolarevicSHuhtaniemiILiuKPDK1 signaling in oocytes controls reproductive aging and lifespan by manipulating the survival of primordial folliclesHum Mol Genet2009182813282410.1093/hmg/ddp21719423553

[B10] ReddyPZhengWLiuKMechanisms maintaining the dormancy and survival of mammalian primordial folliclesTrends Endocrinol Metab2010219610310.1016/j.tem.2009.10.00119913438

[B11] AdhikariDZhengWShenYGorreNHämäläinenTCooneyAJHuhtaniemiILanZJLiuKTsc/mTORC1 signaling in oocytes governs the quiescence and activation of primordial folliclesHum Mol Genet20101939741010.1093/hmg/ddp48319843540PMC2798719

[B12] Li-PingZDa-LeiZJianHLiang-QuanXAi-XiaXXiao-YuDDan-FengTYue-HuiZProto-oncogene c-erbB2 initiates rat primordial follicle growth via PKC and MAPK pathwaysReprod Biol Endocrinol20108667410.1186/1477-7827-8-6620565902PMC2903600

[B13] Talmor-CohenATomashov-MatarREliyahuEShapiroRShalgiRAre Src family kinases involved in cell cycle resumption in rat eggs?Reproduction200412745546310.1530/rep.1.0010415047936

[B14] RobyKFSonDSTaylorCCMontgomery-RiceVKirchoffJTangSTerranovaPFAlterations in reproductive function in SRC tyrosine kinase knockout miceEndocrine20052616917610.1385/ENDO:26:2:16915888929

[B15] LuriaATennenbaumTSunQYRubinsteinSBreitbartHDifferential localization of conventional protein kinase C isoforms during mouse oocyte developmentBiol Reprod2000621564157010.1095/biolreprod62.6.156410819756

[B16] LuQSmithGDChenDYYangZHanZMSchattenHSunQYPhosphorylation of mitogen-activated protein kinase is regulated by protein kinase C, cyclic 3',5'-adenosine monophosphate, and protein phosphatase modulators during meiosis resumption in rat oocytesBiol Reprod2001641444145010.1095/biolreprod64.5.144411319150

[B17] MengXQZhengKGLiYLRole of Src family kinases in oocytes meiosis maturity and fertilization of mice and ratsJ Reprod Contracept2007276164

[B18] JinXHanCSZhangXSYuanJXHuZYLiuYXSignal transduction of stem cell factor in promoting early follicle developmentMol Cell Endocrinol200522931010.1016/j.mce.2004.10.00615607523

RETRACTED

[B19] SeraficaMDGotoTTrounsonAOTranscripts from a human primordial follicle cDNA libraryHum Reprod2005202074209110.1093/humrep/dei03015845590

[B20] FaergeITerryBKalousJWahlPLesslMOttesenJLHyttelPGrøndahlCResumption of meiosis induced by meiosis-activating sterol has a different signal transduction pathway than spontaneous resumption of meiosis in denuded mouse oocytes cultured in vitroBiol Reprod2001651751175810.1095/biolreprod65.6.175111717137

[B21] Talmor-CohenAEliyahuEShalgiRSignalling in mammalian egg activation: role of protein kinasesMol Cell Endocrinol200218714514910.1016/S0303-7207(01)00691-811988322

[B22] FanHYTongCLiMYLianLChenDYSchattenHSunQYTranslocation of the classic protein kinase C isoforms in porcine oocytes: implications of protein kinase C involvement in the regulation of nuclear activity and cortical granule exocytosisExp Cell Res200227718319110.1006/excr.2002.554712083800

[B23] ThamilselvanVCraigDHBassonMDFAK association with multiple signal proteins mediates pressure-induced colon cancer cell adhesion via a Src-dependent PI3K/Akt pathwayFASEB J2007211730174110.1096/fj.06-6545com17317726

[B24] FukuiYHanafusaHRequirement of phosphatidylinositol-3 kinase modification for its association with p60srcMol Cell Biol19911119721979184866610.1128/mcb.11.4.1972-1979.1991PMC359882

[B25] HaefnerBBaxterRFinchamVJDownesCPFrameMCCooperation of Src homology domains in the regulated binding of phosphatidylinositol 3-kinase. A role for the Src homology 2 domainJ Biol Chem19952707937794310.1074/jbc.270.14.79377713890

[B26] MartinGSThe hunting of the SrcNat Rev Mol Cell Biol2001246747510.1038/3507309411389470

[B27] TaylorSJShallowayDAn RNA-binding protein associated with Src through its SH2 and SH3 domains in mitosisNature199436886787110.1038/368867a07512694

[B28] AlexandropoulosKBaltimoreDCoordinate activation of c-Src by SH3- and SH2-binding sites on a novel p130Cas-related protein, SinGenes Dev1996101341135510.1101/gad.10.11.13418647432

[B29] BurnhamMRBruce-StaskalPJHarteMTWeidowCLMaAWeedSABoutonAHRegulation of c-Src activity and function by the adapter protein CASMol Cell Biol2000205865587810.1128/MCB.20.16.5865-5878.200010913170PMC86064

[B30] SatoKIwasakiTHiraharaSNishihiraYFukamiYMolecular dissection of egg fertilization signaling with the aid of tyrosine kinase-specific inhibitor and activator strategiesBiochim Biophys Acta2004169710312110.1016/j.bbapap.2003.11.01715023354

[B31] ZhengKGMengXQYangYYuYSLiuDCLiYLRequirements of Src family kinase during meiotic maturation in mouse oocyteMol Reprod Dev20077412613110.1002/mrd.2061316941660

[B32] KidderGMMhawiAAGap junctions and ovarian folliculogenesisReproduction200212361362010.1530/rep.0.123061312006089

RETRACTED

[B33] RobyKFSonDSTaylorCCMontgomery-RiceVKirchoffJTangSTerranovaPFAlterations in reproductive function in SRC tyrosine kinase knockout miceEndocrine20052616917610.1385/ENDO:26:2:16915888929

[B34] SunQYLuQBreitbartHChenDYcAMP inhibits MAP kinase activation and reinitiation of meiosis, but exerts no effects after germinal vesicle breakdown (GVBD) in mouse oocytesReprod Fertil Dev199911818610.1071/RD9903810735551

